# Blockchain-Based Supply Chain System for Olive Fields Using WSNs

**DOI:** 10.1155/2022/9776776

**Published:** 2022-09-23

**Authors:** Oussama Ghorbel, Tarek Frikha, Abir hajji, Raed Alabdali, Rami Ayadi, Mohamed Abbas Elmasry

**Affiliations:** ^1^Department of Computer Science, Jouf University, Sakakah, AlQurayat Region, Saudi Arabia; ^2^CES-Lab, Sfax University, Sfax, Tunisia; ^3^Gabes University, Gabes, Tunisia; ^4^National Egyptian E-Leaning University (EELU), Giza, Egypt

## Abstract

The agricultural domain in developing countries is mostly dictated by archaic rules based on traditions and inherited practices. With the evolution of digitalization and technology, it seems essential to apply new technologies to the agricultural field. Among the technologies to be exploited in agriculture, we mention sensors, IoT, WSN, cloud, blockchain, etc. We talk about smart agriculture in this case. In this paper, we propose a platform secured by blockchain for monitoring and securing production. This platform uses IoT connected sensors to track and save data. Our system is used to monitor the production process of olive trees. The goal is to track everything that enters and leaves our olive tree production from fertilizers, insecticides, and fortifiers to olives, trimming etc. The blockchain via its decentralized system allow a secure, irreversible, and clear monitoring. A dashboard allow us to highlight the changes while facilitating the work of farmers. Our prototype will be embedded via a Raspberry Pi 4 platform.

## 1. Introduction

Using deep learning, machine learning, cloud, 4G, etc., it is becoming a common practice not only in technology fields such as IT, security, surveillance but also industry, transportation, e-health, smart cities, etc. Among the fields that need this evolution, we can also mention agriculture. The use of data and information has become increasingly crucial for the agricultural sector to improve productivity and sustainability. Internet of Things (IoT) technologies [1, 2] significantly increase the effectiveness and efficiency of data collection, storage, analysis, and use in agriculture. It allows farmers especially and the agricultural community more generally to easily obtain updated information and thus make better decisions in their daily farming.

For example, remote sensing data [3] on soil conditions can help farmers manage their crops, and the collected data can be accessed via the web or cell phones. This reduces the cost of information and thus facilitates farmers' access to markets and financial assistance. The development of the Global Positioning System (GPS) facilitates file mapping, machine guidance, and crop tracking. To enable the supply chain and minimize the risk of errors, fraud, and theft, blockchain technology is used. This technology is based on distributed registers [4, 5]. The use of blockchain is not only related to cryptocurrency (Bitcoin, Ethereum, etc.) but also other sectors that are starting to work on concrete use cases include industry via Industry 4.0 & 5.0 [6], e-health [7–9] such as medical records tracking and EHR [7, 10], paramedical and sports applications [2], and smart cities [11, 12].

In this paper, we propose an embedded agricultural system for monitoring an olive field based on IoT managed by a decentralized blockchain-based system guaranteeing the reliability of data provided by various sensors. We will highlight the practical case of smart and water efficient irrigation system based on wireless sensor networks and secured by blockchain.

This paper is organized as follows: We present a state of the art with a definition of blockchain;

In part 2, we present our application scenario and system model; in part 3, we present our simulation; finally, we conclude this paper with a conclusion and future work.

## 2. Related Works

In this section, we discuss four classes of applications in the agricultural sector.

Agri-food production and supply chains [13–16] have been the subject of many studies. Indeed, using the technological evolution has allowed to fully improve the productivity. Li et al. [17] developed a dynamic planning method for the agri-food supply chain. As a result, they were able to maximize production, increase profiles, and decrease any waste.

Dey et al. [18] developed a Food-SQRBlock (Food Safety Quick Response Block) blockchain using blockchain and QR codes. They also proposed a large-scale cloud integration of the developed system to demonstrate the practicality and scalability of the framework along with supporting experimental evaluation.

While the majority of the work is used to track the supply chain, some have used the blockchain as an electronic money system and particularly as an electronic currency. In Ref. [19], Foroglou and Tsilidou have used the blockchain not only to implement a payment platform but also as a system for managing contracts, voting, property rights etc.

In Ref. [20], Tian proposed a theoretical real-time food traceability system using HACCP system, blockchain, and IoT. The authors claimed to be able to achieve transparency, reliability and security with the proposed model but did not provide an experimental implementation and evaluation of the system. Leng et al. [21] introduced a dual-chain based agricultural supply chain architecture using a public blockchain. They also studied storage mode, resource rent seeking, and consensus algorithms but did not assess the speed and skill of consensus algorithms considering the case of a large number of nodes and resources on the platform. In addition, access management for the user should be further investigated.

Surasak et al. [22] presented an IoT-based blockchain traceability system particularly designed for Thai agricultural products. Blockchain was used to create a distributed ledger to increase data integrity and transparency and a Structured Query Language (SQL) database was used to make the platform user-friendly. Further research on the integration of blockchain into the proposed system is needed to improve the efficiency of the system. Blockchain was used to create a distributed ledger to increase data integrity and transparency and a Structured Query Language (SQL) database was used to make the platform user-friendly. Further research on the integration of blockchain into the proposed system is needed to improve the efficiency of the system. Blockchain was used to create a distributed ledger to increase data integrity and transparency, and a Structured Query Language (SQL) database was used to make the platform user-friendly. Further research on the integration of blockchain into the proposed system is needed to improve the efficiency of the system.

Dakshayini and Prabhu. [23] proposed a blockchain, big data, and cloud-integrated crop monitoring system that attempts to realize effective demand-based decision support and achieve a simple, verifiable, and efficient system. The authors also proposed a crop exchange platform to sell the agri-products at different stages. However, they did not implement the IoT-based blockchain architecture to collect the actual field parameter data and then model the Big Data model.

The use of blockchain is not only applicable to agriculture (vegetables, fruits, etc.) [24] but private blockchain has also been used to track and secure dairy products. Rouaghi uses Hyperledger Fabric blockchain for product tracking [25].

In this paper, we present a system allowing not only to make the supply chain but also to manipulate all the data related to the olive trees such as the inputs (plants, fertilizers, insecticides, water, irrigation etc) but also the harvest (olive, trimming, etc). In this paper, we will propose a platform that uses different sensors, wireless sensor networks, blockchain, cloud etc.

## 3. Materials and Methods

### 3.1. Blockchain Choice

The concept of blockchain can be defined as a decentralized and distributed ledger to store time stamped transactions between many computers in a peer-to-peer network [2]. Thus, any record involved cannot be altered retroactively. This allows blockchain users to audit and verify transactions independently and transparently. Thus, the blockchain consists of blocks, which are connected using cryptographic techniques [26]. Each block must have a hash code of the previous block; a timestamp is a set of confirmed transactions.  Figure 1 illustrates the blockchain.

We can subdivide our blockchain into three types: public, private and permissioned.

#### 3.1.1. Public Blockchain

Public blockchain is an open blockchain. Everyone can access the private blockchain. Bitcoin blockchain operated continuously since its inception. All operate with the support of its public participants [27]. Thus, Bitcoin is the quintessential example of a public blockchain. Anyone can join and leave at their own will.

The various blocks of transactions and the blockchain are public and observable even if the participants are anonymous.

#### 3.1.2. Private Blockchain

Moving on to a private blockchain, access to the blockchain is restricted to selected participants such as participants within an organization.

This restriction helps to simplify normal operations such as block creation and contingency model.

#### 3.1.3. Permissioned Blockchain

The third classification of blockchain is permissioned blockchain, also known as consortium blockchain. It is intended for a consortium of collaborating parties to conduct transactions on blockchain to facilitate governance, provenance, and accountability [28].

Examples include a consortium of all automotive companies, healthcare organizations, industry 4.0, smart agriculture, etc.

Permissioned blockchain has the advantages of a public blockchain by only allowing users with permission to collaborate and transact.

In this paper, we designed an integrated IoT-blockchain architecture, and we choose Ethereum as a type of blockchain for a decentralized agricultural system. We chose Ethereum because it is a permissioned blockchain that can be private or public. It can also execute smart contracts.

To create and maintain our Blockchain Ethereum network, Raspberry Pi 4 and 4 Go are used as it offers low-power consumption and simplicity of their interfaces.

The objective is to set up a platform to monitor the agricultural field, thus, appealing to the IoT on the basis of a blockchain platform. The reasons for setting up this platform are as follows:

- The importance of data confidentiality and the security aspect of agricultural information is justified by blockchain use.
- The need for large volumes of data shows the need to use big data. PoW maintains the security layer of data.
- The need to use data collected in real time from IoT sensors allows information to be updated in real time.

To improve the production result without making our solution complex and with highly consumption, we use the wireless sensor network which will be described in the next part. This WSNs field is considered the best solution to have data from different sensors to make our solution better.

## 4. Wireless Sensor Network

Wireless sensor network has been a growing interest in the scientific and industrial communities, thanks to innovations that have occurred during the last decades in the domains of microelectronics, MEMS (Microelectromechanical system) design, energy harvesting, and wireless technologies [29]. These wirelessly connected sensor networks consist of a large number of sensing nodes densely deployed in the wanted region. These sensing embedded elements are connected to each other through wireless links and work together to collect large amounts of high-fidelity information about different locations, processing them, and transmitting data to gateway nodes also known as sink points. Recent deployments have demonstrated their utility in various domains as described in Figure 2. WSNs are usually used in military operations [30]. Recently, a new set of possible applications has been an active subject of research, such as structural health monitoring [31–33], environmental monitoring [34, 35], agriculture [36], and industrial applications [37–39]. Recent experimentations are currently exploding in terms of usage and performances to improve the way of working in many contexts like automation smart cars to reduce the number of crashes and home automation. The quality of data collected by WSNs has been often unreliable and inaccurate because of the WSN's imperfect nature. Nonetheless, sensor nodes have stringent resource constraints such as memory capacity, computational complexity, and communication bandwidth, and energy consumption. These limited resources make the data generated by the sensor contaminated by noise, obvious error, missing data, duplicated values, and conflicting information. Furthermore, WSNs frequently utilize a large number of sensor nodes in harsh and hostile environments where sensor nodes are vulnerable to malicious attacks; hence, data generated and processed will be controlled by enemies.

### 4.1. Development of the Smart Water Irrigation System with Moisture Monitoring

In our work, we have developed a water-saving irrigation control system that is based on wireless sensor networks [40], whereby the system comprises low-power wireless sensor nodes that communicate through an adhoc ZigBee network. We will monitor soil moisture information parameters such as soil water degree, temperature, and relative humidity that can all be used to measure moisture potential. A four-channel temperature and humidity transmitter will be used to collect this data. The information details are determined by using the various component of the sensor. In the following subsections, we will describe in detail the proposed design.

### 4.2. Smart Water Irrigation System for Farmers

As shown in Figure 3, our system of agriculture irrigation is based on famous technology entitled WSN is made up of four components: an irrigation controller, receiving sensors, a set of sensors, and a network of irrigation pipes. To construct an irrigation node group, sensor nodes that bear soil moisture are disseminated in accordance with the planting and irrigation status of farming. Each node is in charge of keeping track of the soil moisture in a certain area.

A standard WSN, utilizing ZigBee technology based on transmitted wireless data, consists of irrigation region and receiving sensors. Wireless multihop is used to transfer sensor data to the receiving node. Our discipline is designed to install a network for an irrigation pipe on the farming area in the irrigation region and an electrical control valve on the pipe to create an automated water-saving irrigation system. If the control of smart water irrigation is adaptable, the total system will be more versatile.

A water-saving irrigation system may be modified based on the original irrigation pipe network. For greater deployment of the irrigation system pipe network and to save money, an electronic control valve can be fitted. The irrigation controller in the WSN coverage region may spray irrigation in specified locations based on sensor data. This system contains a specific module taking in charge of network supervision. The proposed Smart Water Irrigation System is mainly dependent on wireless sensors networks and water pipeline.

### 4.3. System Hardware Structure

In this part, the hardware structure of the sensor node implemented in the proposed architecture is addressed and illustrated in Figure 4. The controller module, sensor module, ZigBee protocol communication module, and solar self-powered module make up the majority of the hardware structure.

The irrigation controller is built using an embedded system development board as the mainboard. The receiving node receives information through a serial connection and processes the control data. The system is very scalable. The WSNs measure of humidity is realized to be five times in minute (on a 12-second cycle) and send the data to the irrigation controller. When the irrigation controller detects that the humidity sensed by the WSN nodes in a specific location is lower than the prescribed value, it activates the irrigation network's electric control valve. The system will start irrigation and close the electric control valve of the pipe network in this region when the soil humidity in the area reaches a particular level.

### 4.4. Proposed Architecture

In this work, we propose the architecture as shown in Figure 5. Thus, the different actors of our agricultural system (farmers, vendors, distributors, etc.) are connected via a wireless sensor network. The data are saved on a database keeping the different traces of each transaction on blockchain. This traceability allows protecting not only all actors but also the plants of our farm.

It is important to point out that the data in the blockchain is encrypted using the Keccak 256 algorithm. This data can only be accessed using the public key of the sender and the private key of the receiver. The data are therefore encrypted and protected.

Each piece of data is encrypted using the receiver's public key and the sender's private key. Thus, only the person who has his private key can open a data encrypted with the public key.

The system uses the PoW as a consensus. Since our blockchain does not use crypto-currencies and does not offer crypto-currencies as an offering for mining, it is therefore difficult to find malicious people who would like to decrypt the transactions or try to steal them. Thus, the security layer used in the blockchain allows having an efficient system for our farming application.

## 5. Obtained Results

In this section, we propose different results obtained after presenting the architecture, as shown in Figure 6. We present two different parts as follows:

- First, the results obtained by the different humidity, temperature, light, and wind sensors as well as the interfaces realized and connected to the blockchain
- Second, a synthesis of the work on irrigation using wireless sensor networks

For example, the rise in temperature can also have contradictory consequences on plants. Thus, the increase in temperature decreases the yield. The use of IoT sensors (temperature, humidity, photoresistor, and wind) in the agricultural field which collects climatic data controls the field and helps producers make the right decisions to improve production.

The temperature and humidity results are shown in Figure 6, while the wind and light curves are shown in Figure 7. The results of our research show that the temperature varies between 0 and 65. Thus, relative humidity (RH) ranges from 0 to 100%. The air is dry when the relative humidity is below 35%. The air is moderately humid between 35% and 65%, and the air is humid at more than 65% relative humidity. Within the same space, the RH varies according to temperature changes; that is, it increases if the temperature drops and decreases if it rises.

For light, it varies between 0 and 100 lux. The light rate varies with temperature. It increases if the temperature increases and vice versa.

Wind speed affects plants. Frequent winds slow down plant growth and cause malformations: inclination of stems, nondevelopment of organs (leaves, buds, etc.).

We propose to break the supply chain management ecosystem using the Ethereum blockchain as follows: Farmers can control the field via a dashboard too and sell directly to consumers, so it can maintain the freshness of the food product, and its prices will be stable.

The data in the block of each transaction is divided into several parts of the block as follows:

- The system where the blockchain works is a server like a database.
- Any valid transaction has been validated by a block regulated by the protocol.
- Each blockchain block contains those as follows:

  Data (timestamp and transaction information),
  Hash (fingerprints of encrypted mathematical transactions),
  Hash is the unique identifier of the block,
  Hash of the previous block.

The Ethereum blockchain offers consumers who can see where the food product comes from, and then farmers can also view and verify the product until it is delivered to the customer based on location, farmer name, delivery date, number of purchases (kg), product type, and price. Here are the actors involved in the Ethereum blockchain.

### 5.1. Farmers

Those who control the field from the IoT sensors on-site produce the food product harvest and sell it in quantity (kilograms) to consumers.

### 5.2. Consumer

The party that buys product from farmers will be consumed or resold.

Here is a comparison between blockchain and the traditional database in all its aspects.

As described earlier, our application is presented in Figure 8 and is based on blockchain technology. We used Ethereum which was installed on the smart platform Raspberry Pi 4. The data captured by the three sensors must be recorded in Raspberry Pi 4 and in the blockchain. The result is displayed in a web page.

The developed application displays a web page identified by the web address 127.0.0.1, which presents a dashboard, as shown in Figure 9. This dashboard allows farmers to control and monitor the temperature values with their humidity and luminosity values for all months of a year. All collected data are stored in the database.

- The temperature is presented by the curve in light pink, where values are set between 13°C and 48°C.
- The humidity is presented by the dark pink curve, where values vary from 4% to 100%.
- The brightness is presented by the dark red color, where values vary from 35,000 Lux up to 120,000 Lux. Since their values are very large, we have divided the brightness values by 1000. In our dashboard, the brightness values are set between 35 Lux and 120 Lux.

## 6. Discussion

Many applications in various industries have used the new technology. As in our work, we focus on the agriculture field to compare related work. For example, Ref. [41] proposed a smart agriculture system, but some have used the sensors with fuzzy logic to present an intelligent sprinkler system, and others have based their approach only on sensors to monitor the condition of the paper. For precision agriculture, the authors in Ref. [40] used sensors and Raspberry Pi to assess soil fertility and productivity. This approach is different to our approach since we used Ethereum. In addition, in our work, we focus on collecting relevant data to control agricultural conditions mainly temperature, humidity, and light. In Ref. [42], authors added consensus mechanisms in electronic agriculture. In Ref. [43], the authors used smart contracts in the green IoT to create agreements. Green IoT helps realize the vision of a green ambient intelligence. There are several concepts of a sustainable green ecosystem with the use of blockchain such as green energy, green IT, and green finance. All can use smart contracts in a green ecosystem. It is an approach that is different from our approach, where they used smart contracts with IoT and our agricultural sensor-based approach with IoT. In addition, the authors in Ref. [44] used smart contracts for the hyperledger blockchain, where our approach is done on the Ethereum blockchain which can be private and/or public. The integration of IoT and blockchain in Ref. [45] offers more decentralization to make information and systems more reliable and stable. In our approach, we are interested in the IoT with a decentralized system based on the blockchain, and we have added sensors for data collection. In Ref. [46], the blockchain is added to solve a lot of the problems, and above all, the trust and security. For our work, our goal is to improve trust between users without a third party and also to get a lot of information remotely without wasting time from sensors [47].

To summarize, our approach is based on a decentralized system with the use of the Ethereum blockchain in the agricultural sector. Various sensors were used to detect data and facilitate work for farmers.  Table 1 below compares the aforementioned related works to our solution [51, 52].

## 7. Conclusions

The objective of this work focuses on the implementation of an intelligent agricultural framework managed by a decentralized system based on blockchain, as it is a new technology characterized by disintermediation in its use, traceability, and transparency of transactions, infeasibility, distribution, resiliency, security of all data, and greater trust. We have used Ethereum as a decentralized type of blockchain. This paper presents the installation of Ethereum on the Raspberry Pi 4; two nodes were created to have a connected and functional multinode Ethereum network. Sensors are used to obtain data for temperature, humidity, wind, and light; all data are stored in the database. Sensors play an essential role in agriculture. They are the key to collecting data more efficiently in order to make the most appropriate decisions.

The connection between the sensors is done using wireless sensor networks. One of the most challenging aspects of wireless sensor networks is their energy efficiency. That is why we propose an efficient way of utilizing the energy of wireless sensor networks for agriculture production. We are particularly interested in various monitoring techniques suitable our supply chain system for the olive field. To provide WSN with an information platform that can support a better role in agricultural production, the proposed model aims to improve on the shortcomings of existing WSN in the context of energy efficiency. So agriculture is a key factor impacting the global economy; therefore, WSN is important.

At the end, based on our solution, we conclude that our system has linked wireless sensor networks and their low-power system with blockchain technology that allows for secure data and tracking to avoid any attempt to steal or usurp data related to products or agriculture.

## Figures and Tables

**Figure 1:** Blockchain illustration.

**Figure 2:** Application area of wireless sensor networks.

**Figure 3:** Smart water irrigation system based on wireless sensor networks.

**Figure 4:** Hardware structure of the sensor node used in the proposed architecture.

**Figure 5:** Proposed architecture.

**Figure 6:** Temperature and humidity curves.

**Figure 7:** Light and wind curves.

**Figure 8:** Final architecture of the agricultural application.

**Figure 9:** Dashboard.

**Table 1:** Comparison with related works.

Reference	Author	IoT	Fuzzy Logic	Sensors	Consensus mechanisms	Rasp. Pi	Smart contracts
[29]	A.H.Gilson (2020)	✗	✗	✓	✗	✓	✗
[30]	Y.Chen (2020)	✗	✗	✓	✓	✗	✗
[31]	M.S.Munir (2019)	✓	✓	✓	✗	✗	✗
[32]	A.N.Putri (2021)	✓	✗	✓	✗	✗	✗
[34]	P.S.Kumar (2020)	✓	✗	✗	✗	✗	✓
[35]	H.K.Ali (2020)	✗	✗	✗	✗	✗	✓
[36]	D.X.Li (2021)	✓	✗	✗	✗	✗	✓
[37]	T.Noshina (2019)	✓	✗	✗	✓	✗	✓
Our approach	(2022)	✗	✗	✓	✓	✓	✓

Blockchain is used in different application areas such as smart cities (smart parking [12, 48], water meter [49, 50], etc.).

## Data Availability

The data used to support the findings of this study are available from the corresponding author upon request.
